# Basal cell carcinoma and squamous cell carcinoma: Comparison of high‐frequency ultrasound and pathology

**DOI:** 10.1111/srt.13897

**Published:** 2024-08-09

**Authors:** Sepideh Keshavarz Valian, Faezeh Khorasanizadeh, Kambiz Kamyab, Sadra Nourazar, Sahar Montazeri, Arghavan Azizpour

**Affiliations:** ^1^ Razi Hospital Tehran University of Medical Sciences Tehran Iran; ^2^ InPedia Association, Students’ Scientific Research Center Tehran University of Medical Sciences Tehran Iran

**Keywords:** high‐frequency ultrasound, malignancy, skin tumor

## Abstract

**Background:**

Skin neoplasms, particularly basal cell carcinoma (BCC) and squamous cell carcinoma (SCC), are prevalent forms of skin malignancies. To enhance accurate diagnosis, non‐invasive techniques including high‐frequency ultrasound (HFUS) are crucial. HFUS offers deeper penetration compared to reflectance confocal microscopy (RCM), and optical coherence tomography (OCT), making it valuable for examining skin structures. The aim of this study was to investigate and diagnose localized manifestation of BCC and SCC with HFUS and compare it with pathology results in patients referred to Razi Hospital, Tehran, Iran.

**Method and materials:**

This study included patients diagnosed with BCC and SCC, with clinical and pathological confirmation, attending the oncology clinic of Razi Hospital, Tehran, Iran, from 2022 to 2023. Exclusion criteria comprised metastatic and recurrent cases, patients who underwent treatment or surgery, and tumors located in anatomically challenging areas. HFUS with a 20 MHz probe and Doppler ultrasound were employed to examine the skin. Tumors were subsequently excised, fixed in formalin, and sent for pathological assessment. Ultrasound findings were compared with pathology results.

**Results:**

The study assessed 40 patients, with half diagnosed with SCC and the other half with BCC. The majority of SCC patients were male (80%), while BCC patients were relatively evenly divided between males (65%) and females (35%). The mean age was 59.15 ± 11.9 years for SCC and 63.4 ± 8.9 years for BCC. Cheeks (20%) and lips (35%) were the most common sampling sites for BCC and SCC, respectively. The correlation coefficients for tumor size and depth between ultrasound and pathology were 0.981 and 0.912, respectively, indicating a high level of agreement between the two methods.

**Conclusion:**

In BCC patients, there was complete agreement between sonographic loco‐regional extension and pathology findings. However, some discordance (30%) was observed in SCC cases. The study demonstrated a strong correlation between ultrasound and pathology in accurately detecting the depth and extent of the tumor. However, due to the inclusion of only patients with positive pathology, it is not appropriate to evaluate the diagnostic test values and compare them with pathology results. Therefore, it is highly recommended to carry out additional studies with larger sample sizes to further validate these findings.

## 1 INTRODUCTION

Skin neoplasms are among the most common malignancies. Malignancies arising from the epidermis include cutaneous melanoma (CM), non‐melanoma cancers, such as basal cell carcinoma (BCC), squamous cell carcinoma (SCC), and Merkel cell carcinoma (MCC). BCC and SCC alone account for 95% of skin malignancies.^1^ Despite being malignant and invasive, BCC is rarely fatal, but it still can invade and damage surrounding tissues, causing significant destruction and disfigurement.^2^, ^3^ SCC is a keratinocyte carcinoma that accounts for at least 20% of skin cancer‐related deaths worldwide and its prevalence is increasing.^4^, ^5^ Compared to BCC, SCC has unique features, including a chronic inflammatory process, rapid growth pattern, poor differentiation, and lymphovascular invasion. Therefore, there is a need for invasive diagnostic methods.

Misdiagnosis of similar malignancies may lead to treatment delays, higher medical costs, and functional and aesthetic complications. Therefore, new diagnostic methods are vital to distinguish high‐risk BCC from SCC. Biopsy is considered the gold standard for differentiating high‐risk BCC from SCC. However, the invasive part of the tumor might be missed because the biopsy only examines a limited area. Additionally, biopsy is invasive and is not able to assess the size, thickness, and penetration depth of the malignancy. Dermoscopy also only provides information about the surface of the tumor and it may miss the infiltrative features that may be present only at the deeper periphery of it. Reflectance confocal microscopy (RCM) and optical coherence tomography (OCT) provide high‐resolution but incomplete information due to their relatively shallow penetration (0.5 mm). Therefore, it is difficult to distinguish high‐risk BCC from SCC.

Due to its high resolution, high‐frequency ultrasound (HFUS) can be used to examine all structures in the skin, including the epidermis, dermis, subcutaneous fat layer, muscle layer, and blood vessels.^6^ It also has higher depth of penetration compared to OCT and RCM and therefore achieves the reasonable balance between resolution and penetration depth that other methods lack. Considering these features and other features such as non‐invasiveness and cost‐effectiveness, HFUS may be a reliable tool to diagnose these two cancers that are similar in appearance.^7^ Also, ultrasound image guided tumor depth is crucial for determining the CORRECT energy for a superficial radiation therapy of these cancers.^8^

In this regard, the aim of this study was to investigate and diagnose localized manifestation of BCC and SCC with HFUS and compare it with pathology results in patients referred to Razi Hospital, Tehran, Iran, in 2022–2023.

### 1.1 Method and materials

In this study, all patients with clinical and pathological diagnosis of BCC and SCC who were referred to the oncology clinic of Razi Hospital, Tehran, Iran, in 2022–2023 (20 SCC patients and 20 BCC patients) were included. The inclusion criteria for this study included clinical confirmation of SCC and BCC by a dermatologist and histological confirmation of BCC and SCC by a pathologist. However, metastatic and recurrent cases, patients who had undergone treatment and surgery (such as cryotherapy), and patients with tumors situated in anatomical regions that rendered it impractical or unfeasible to position the ultrasound probe were excluded.

Initially, the patients underwent dermoscopy. The investigation for BCC involved examining various factors, including the tumor's size, pigment presence, arborizing vessel, maple leaf‐like area, blue gray ovoid nests, and spoke wheel structure. Additionally, the presence of keratin and scale, blood spots, hairpin vessels, white circle, linear and irregular vessels were also examined for SCC.

The skin was examined using HFUS with a 20 MHz probe, and Doppler ultrasound was conducted. Due to maximum penetration of 6 mm with the 20 MHz probe, a variable depth probe with 13–18 MHz was used to investigate infiltrative BCCs and aggressive SCCs.^8^ Importantly, the radiologist was uninformed about the pathology results.

The ultrasound examination included measurements of various characteristics such as tumor type, shape, location, composition (solid or cystic), echogenicity (hypoechoic for solid and anechoic for cystic), homogeneity, extent of invasion, vascularity type and location, and the thickness of the malignancy. Additionally, locoregional expansion around the malignancy was also assessed.

Subsequently, the tumor was removed with a margin of 4 mm, which was then placed in formalin and sent to the pathologist. The pathologist conducted an assessment of the histopathological findings, encompassing tumor type, marginal manifestations, depth of the lesion, and invasion. Importantly, the pathologist was unaware of the ultrasound results during this evaluation. Ultimately, a comparison was made between the ultrasound and pathology findings.

## 2 RESULTS

In this study, 40 patients were examined, 20 (50%) of whom were diagnosed with SCC and 20 (50%) with BCC. Of the 20 people with SCC, 16 were male (80%) and 4 (20%) were female, while in BCC patients, 13 were male (65%) and 7 were female (35%). The mean age of the referring patients with SCC and BCC was 59.15 ± 11.9 and 63.4 ± 8.9 years, respectively.

Sampling from different areas was performed as demonstrated in Table 1. In BCC and SCC patients, most samples were taken from the cheek (five cases, 20%), and the lip (seven cases, 35%), respectively.

**TABLE 1:** Laboratory findings of SCC and BCC patients.

	SCC	BCC
Sex		
Male	16 (80)	13 (65)
Female	4 (20)	7 (35)
Mean age	59.15 ± 11.9	63.4 ± 8.9
Sonographic locoregional extension	14 (70)	20 (100)
Affected periphery	20 (100)	20 (100)
Sampling site distribution		
Eye	1 (5.2)	3 (17.6)
Ear	1 (5.2)	2 (11.7)
Vortex	0 (0)	1 (5.8)
Scalp	4 (21.0)	2 (11.7)
Neck	0 (0)	1 (5.8)
Lip	7 (36.8)	0 (0)
Thigh	0 (0)	1 (5.8)
Parietal scalp	0 (0)	1 (5.8)
Occipital scalp	0 (0)	1 (5.8)
Nose	1 (5.2)	2 (11.7)
Calf	3 (15.7)	0 (0)
Forehead	1 (5.2)	1 (5.8)
Cheek	2 (10.5)	5 (29.4)
Vascular intensity		
Neg	2 (10)	3 (15)
1+	6 (30)	12 (60)
2+	8 (40)	5 (25)
3+	4 (20)	0 (0)
Dermoscopic characteristics		
Arborizing vessel		
Pos	–	18 (90)
Neg	–	2 (10)
Blue Gray Ovid Nest		
Pos	–	10 (50)
Neg	–	10 (50)
Spoke wheel		
Pos	–	9 (45)
Neg	–	11 (55)
Maple Leaf Like		
Pos	–	17 (85)
Neg	–	3 (15)
Scale keratin		
Pos	18 (90)	–
Neg	2 (10)	–
Blood spot		
Pos	9 (45)	–
Neg	11 (55)	–
White circle		
Pos	16 (80)	–
Neg	4 (20)	–
Hairpin vessel		
Pos	11 (55)	–
Neg	9 (45)	–
Irregular linear vessel		
Pos	5 (25)	–
Neg	15 (75)	–

Eighteen patients with BCC (90%) and 13 patients with SCC (65%) exhibited a high risk of recurrency. In our study, 19 cases of BCC patients and 17 cases of SCC patients were exposed to ultraviolet rays.

All cases of BCC and SCC were confirmed by pathology. Nineteen cases of SCC patients (95%) and 16 cases of BCC patients (80%) were correctly diagnosed by ultrasound. Based on the ultrasound results, no notable correlation was found between tumor type and tumor vascularity (*p* = 0.6). Table 1 illustrates the vascular intensity of tumors observed in the ultrasound scans of patients diagnosed with BCC and SCC.

For BCC patients the arborizing vessel, ovid nest blue gray, spoke wheel, and maple Leaf like characteristics were analyzed. Scale and keratin, blood spot, white circle, hairpin Vessel, irregular and linear vessel were also examined in SCC patients using dermoscopy (Table 1).

For all patients diagnosed with BCC, the sonographic locoregional extension matched the reported affected periphery on pathology in every case. However, there was a mismatch between sonographic findings and pathology margin in 30% of SCC cases (six patients).

Table 2 indicates the reported findings regarding tumor size, including transverse diameter and depth diameter, in patients diagnosed with BCC and SCC. These measurements were obtained using pathology and ultrasound methods. Both methods show higher average transverse diameter and depth diameter in SCC patients.

**TABLE 2:** Transverse and depth diameter in pathology and ultrasound methods.

	Transverse diameter		Depth diameter	
	Pathology	Ultrasound	Pathology	Ultrasound
SCC				
Mean	19.6400	20.0300	4.4950	5.2170
95% confidence interval for mean				
Lower bound	14.0803	3.2901	3.2901	3.2901
Upper bound	25.9797	7.1439	7.1439	7.1439
5% Trimmed Mean	18.8611	19.1111	3.9444	4.8300
Median	14.6000	15.9500	2.4000	3.7500
Variance	174.506	161.610	16.487	16.951
Std. deviation	13.21006	12.71258	4.06040	4.11722
Minimum	4.30	5.60	1.10	1.60
Maximum	49.00	51.00	17.80	15.80
Range	44.70	45.40	16.70	14.20
Interquartile range	19.63	18.13	4.53	4.53
BCC				
Mean	13.3500	13.4850	3.1700	3.4900
95% confidence interval for mean				
Lower bound	9.0168	2.5273	2.5273	2.5273
Upper bound	17.9532	4.4527	4.4527	4.4527
5% Trimmed mean	12.1000	12.0667	3.0389	3.3611
Median	11.5000	11.6000	2.5500	2.6500
Variance	87.748	91.147	4.399	4.231
Std. deviation	9.36738	9.54707	2.09739	2.05705
Minimum	3.20	3.50	0.70	1.00
Maximum	46.00	49.00	8.00	8.30
Range	42.80	45.50	7.30	7.30
Interquartile range	9.48	8.28	3.40	3.35

The correlation coefficient between the size of the tumor in ultrasound and pathology was 0.981 and the correlation coefficient between the depth of the tumor in ultrasound and pathology was 0.912, indicating that there is a high agreement between the results of these two tests (Figures 1 and 2).

**FIGURE 1:** Correlation between lesion size in ultrasound and pathology.

**FIGURE 2:** Correlation between lesion depth in ultrasound and pathology.

## 3 DISCUSSION

This study involved the examination of 20 patients with SCC (50%) and 20 patients with BCC (50%). Among the 20 individuals with SCC, 16 were male (80%) and 4 (20%) were female. In the group of BCC patients, 13 were male (65%) and 7 were female (35%). The analysis did not reveal any significant statistical difference in terms of gender (*p* = 0.48). The average age of the patients with SCC and BCC was 59.15 ± 11.9 and 63.4 ± 8.9 years, respectively. There was no statistically significant difference observed in terms of age (*p* = 0.2). However, in the study of Emadian et al. conducted in Iran, there was a significant relationship between the age of patients and the prevalence of SCC (*p* = 0.40).^8^ In the report of Mirzaei et al. in Tehran province, the incidence of skin cancer increased in both sexes with increasing age.^9^

There was no statistically significant difference in gender between high‐risk BCC and SCC groups (*p* = 0.135). However, the 2018 Que study supports a male predominance in the incidence of SCC.^10^ Furthermore, there was a statistically significant difference in age (*p* < 0.001). The median age of SCC patients was reported to be 79.5 years, while the median age of high‐risk BCC patients was 68.0 years.^11^

In our study, the most common sampling sites were cheeks in BCC patients (five cases, 20%) and lips in SCC patients (seven cases, 35%). In a previous study conducted in Iran, lip was the most common site of manifestation in SCC skin malignancies. In other studies, the most common site of SCC manifestation in the face of people exposed to sunlight was the lower lip, which is mainly due to the formation of actinic cheilitis in the lower lip.^12^ It was also found that both high‐risk BCC and cSCC lesions were mainly located in UV‐irradiated sites, which is consistent with a previous study.^13^

Chen's study in 2022 found no significant disparity between the two groups concerning tumor shape, tumor margin, layer involvement, pseudopodia, and suspected lymph node involvement.^11^ However, it was observed that cSCC tumors tended to be larger and thicker than high‐risk BCC tumors. This finding is consistent with a previous study that reported the majority of cSCC lesions to be thicker than 2.0 mm,^14^ while high‐risk BCC lesions were not more than 2.01 mm thick.^15^ In our study, the thickness of high‐risk BCC and SCC lesions was measured as 3.8 ± 2.3 and 5.6 ± 4.2 mm, respectively.

The ultrasound findings in our study showed that 95% of patients with SCC and 85% of patients with BCC had positive tumor vascularity, with no significant correlation between disease type and tumor vascularity (*p* = 0.6). Jambusaria‐Pahlajani study found that SCC and BCC lesions both exhibit high levels of blood flow.^16^ Likewise, Vega et al. suggested that BCC lesions with higher vascularity in BCC lesions indicates a more aggressive subtype.^17^ On the other hand, it was observed that hypervascularity can be seen in cSCC lesions. Therefore, it is difficult to diagnose these two diseases based on the frequency of blood flow.

All patients with BCC had negative results for ultrasound leucorginal spread, while 70% of patients with SCC had negative results and 30% had positive results. This difference was statistically significant with a *p*‐value of 0.02. The sonographic leucorginal extension matched the pathology margin in all patients with BCC, but in 30% of patients with SCC, there was a discrepancy between the two.

HFUS can detect various internal characteristics of high‐risk BCC and cSCC, including lesion size, thickness, hyperechoic points in posterior acoustic shadowing, and Doppler vascularity pattern. By utilizing these features, a diagnostic model can be developed to differentiate high‐risk BCC from cSCC. Thus, HFUS can play a crucial role in distinguishing between high‐risk BCC and cSCC.^11^ Additionally, previous studies have proved that ultrasound guided depth determination is in good concordance with MRI radiologic evaluation (a gold standard).^18^

In Nasiri Kashani's study in Iran, the average tumor depth in HFUS (1353.68 ± 656.456 microns) was lower than the value measured by the dermatologist (1560.71 ± 1044.323 microns). But this difference was not statistically significant. The mean diameter of the largest tumor in HFUS and pathology was 5996.77 ± 2271.783 and 3891.07 ± 1995.4 microns, respectively (*p* < 0.001). There was a low correlation in diameter (*r* = 0.27, *p* < 0.05) and a moderate correlation in depth (r = 0.45, *p* < 0.001) in BCC patients between the two methods.^19^ In our study, the correlation coefficient between the size of the tumor in ultrasound and pathology was 0.981 and the correlation coefficient between the depth of the tumor in ultrasound and pathology was 0.912, both indicating that there is a high agreement between the results of these two tests. Our results were in concordance of previous studies.^20^

## 4 CONCLUSION

In our study, the most frequently observed dermoscopy finding in patients with BCC was arborizing vessel, reported in 90% of cases, followed by leaf like blue, reported in 85% of cases. Additionally, in cases of SCC, scale‐Keratin and white circle were reported in 90% and 80% of cases, respectively. Sonographic locoregional extension was completely consistent with the affected periphery reported on pathology in patients with BCC (100%), while discordance was reported in 30% (six patients) with SCC. A high correlation between two methods of ultrasound and pathology was seen in detecting the depth and extent of the tumor. Since all patients with positive pathology were included in this study, it would be unreasonable to assess the diagnostic test values and compare them with pathology results. Hence, it is advisable to conduct further studies with larger sample sizes.

## CONFLICT OF INTEREST STATEMENT

None to declare.

## Data Availability

Data is available on request due to ethical/privacy restrictions.
